# Automated Recognition of Cancer Tissues through Deep Learning Framework from the Photoacoustic Specimen

**DOI:** 10.1155/2022/4356744

**Published:** 2022-08-10

**Authors:** Gayathry Sobhanan Warrier, T. M. Amirthalakshmi, K. Nimala, T. Thaj Mary Delsy, P. Stella Rose Malar, G. Ramkumar, Raja Raju

**Affiliations:** ^1^Department of Computer Science and Engineering, SCMS School of Engineering and Technology, Ernakulam 683576, Kerala, India; ^2^Department of Electronics and Communication Engineering, SRM Institute of Science and Technology, Ramapuram, Chennai 600089, Tamil Nadu, India; ^3^Department of Networking and Communications, SRM Institute of Science and Technology, SRM Nagar, Kattankulathur, Chennai 603203, Tamil Nadu, India; ^4^School of Electrical and Electronics, Sathyabama Institute of Science and Technology, Chennai 600119, Tamil Nadu, India; ^5^Department of Electronics and Communication Engineering, JP College of Engineering, Tenkasi 627852, Tamil Nadu, India; ^6^Department of Electronics and Communication Engineering, Saveetha School of Engineering, SIMATS, Chennai 602105, Tamil Nadu, India; ^7^Department of Mechanical Engineering, St. Joseph College of Engineering and Technology, St. Joseph University in Tanzania, Dar es Salaam, Tanzania

## Abstract

The fast advancement of biomedical research technology has expanded and enhanced the spectrum of diagnostic instruments. Various research groups have found optical imaging, ultrasonic imaging, and magnetic resonance imaging to create multifunctional devices that are critical for biomedical activities. Multispectral photoacoustic imaging that integrates the ideas of optical and ultrasonic technologies is one of the most essential instruments. At the same time, early cancer identification is becoming increasingly important in order to minimize fatality. Deep learning (DL) techniques have recently advanced to the point where they can be used to diagnose and classify cancer using biological images. This paper describes a hybrid optimization method that combines in-depth transfer learning-based cancer detection with multispectral photoacoustic imaging. The goal of the PS-ACO-RNN approach is to use ultrasound images to detect and classify the presence of cancer. Bilateral filtration (BF) is often used as a noise removal approach in image processing. In addition, lightweight LEDNet models are used to separate the biological images. A feature extractor with particle swarm with ant colony optimization (PS-ACO) paradigm can also be used. Finally, biological images assign appropriate class labels using a recurrent neural network (RNN) model. The effectiveness of the PS-ACO-RNN technique is verified using a benchmark database, and test results show that the PS-ACO-RNN approach works better than current approaches.

## 1. Introduction

Cancer had been recognized as a leading cause of mortality in both industrialized and developed economies; as a result, the GLOBOCAN and American Cancer Association approximate the amount of new cancer-related mortality every year and compile their most up-to-date data on inhabitants' cancer rates. As per the estimate, by 2020, the United States would have 606,520 cancer sufferers and 1,806,590 new cancer sufferers. The percentage of patients grows as they get older. However, early detection can boost breast survival rates by up to 80%. As a result, there is a pressing need to enhance diagnostics in order to achieve successful timely detection. Microscopic image analytical techniques, such as particular cell counts, cell shape, cell location, and cell classification, have been widely employed for biomedical research and illness detection for generations. Microscopic imaging of cellular components, in particular, aids in the confirmation of the existence of certain illnesses, tumor classification, and the understanding of cell genetic and molecular systems. Over past 50 years, though, misauthentication of cell cultures based on the cross has been recognized as a severe concern. In principle, inaccurate labeling, sharing of cell culture media, and cross-use of pipette tips can lead to cross-contamination of tumor cell lines [1].

PCLs are identified in the clinical setting by visually inspecting pictures from magnetic resonance imaging (MRI), endoscopic ultrasonography (EUS), or computed tomography (CT). EUS is one of these imaging techniques that produces a high-resolution image and allows for repeated treatments such as nonionizing imaging. Furthermore, the definitive diagnosis of MRI and CT in the diagnosis of PCLs has been described to be 39–50% and 40–44%, respectively. EUS has a diagnostic accuracy of about 95% for PCLs that are malignant or premalignant. Operators of EUS processes, on the other hand, must have extensive working qualifications as well as advanced technological skills. Clinicians should execute at least 150 supervised instances to gain comprehensive competency in all areas of EUS. As a consequence, an operator with limited expertise may misdiagnose patients, and even a seasoned expert could be influenced by tiredness and negligence as a result of long-term EUS operations. A computer-aided diagnosis system (CAD) was recently established to support doctors in the diagnostic medical pictures, following recent improvements in artificial intelligence and digital imaging processing. Another function of the CAD system is to locate the image's region of interest (ROI). The ROIs are dynamically separated from other regions in medical pictures when differentiation in the tumors is detected. A condition is diagnosed by analyzing the properties of the ROI using the segmentation results [2].

Since it is the inherent molecular vibrations that examine the chemical components of the substance, this defining the appropriate of the substance is accomplished without even any stain or extra treatment. FTIR photography could be used to explore the tissue's geographic coverage since it retains the histological properties of tissue samples even while allowing for the detection and characterization of molecular biochemical. This method automates a component of research aimed at investigating malignancies, reducing inter and intraobserver participation in prognostic and treatment decisions, while freeing pathologists from heavy daily labor. Alternative histological recognition systems could significantly reduce workload, provide quality assurance, and lower expenses. Unfortunately, there seems to be no simple technique to assist pathologists in this work, and no clinical equipment is presently available for regular usage. As a result, high-throughput, computerized, and objective techniques for prostate pathologies are required in both clinical and research settings. A manual pattern matching procedure that compares features in the tissue sample to requirements specified is used to identify structural aberrations suggestive of disease. Human beings are capable of recognizing illness from a broad realm of the everyday and disease stages, overcoming confounding artefacts, detecting exceptional instances, and even recognizing diagnostic flaws because of manual inspection. However, manual inspection takes time and frequently results in differences in disease classification [3].

Due to the necessity for objectivation and quantification of these pathogenic factors, spectroscopic methods, particularly Fourier transform infrared (FTIR) spectroscopy, have reawakened attention. Depending on the absorbance of IR light by vibrational transitions in hydrogen bonding, FTIR spectroscopy produces distinctive spectrum patterns that are linked to the chemical nature and orientation of the components in the sample through intricate interactions. The FTIR spectrum is responsive to the chemical composition because the energy required for a vibrational or rotation transformation is largely reliant on the chemical reactions microenvironment. As a result, distinctive frequency components could be linked to sample biological properties. This distinctive identity of the material is achieved without any staining or further preparation because it is the intrinsic molecule oscillations that explore the chemical components of the material. Because FTIR imaging preserves the histopathological characteristics of the tissue sections while simultaneously providing the identification and quantification of chemical biochemistry, it can also be used to investigate the tissue's geographic diversity. This technique has the ability to automate a portion of the pathologic evaluation of malignancies, limiting inter- and intraobserver involvement in diagnostic and prognostic judgments while also relieving pathologists of the large daily workload. Moreover, because biological changes in cellular membranes usually occur before morphological features, which have been the basis of histopathological assessment, FTIR scanning may possibly alter the assessment of many pathologic characteristics by collecting spatially distributed high-quality data [4].

Photoacoustic imaging (PAI) is a nonionizing, noninvasive multimodal imaging technique that has advanced significantly over the years, to the point where clinical trials are becoming a viable option. PAI advantages by both rich and adaptable optical contrasts and excellent (diffraction-limited) positional accuracy related to low-scattering ultrasound waves transmission due to its hybrid character, that is, optical stimulation and acoustic detecting. By using electromagnetic energy generated ultrasonic vibrations as a transport to gather absorption spectra information of tissue, photoacoustic photography goes through the dispersion limitation of high-resolution optical imaging (1 mm). PAI is a comparatively recent imaging technique that could efficiently realize the structural or functional characteristics of living tissues, making it a potent image technique for researching physiological, pathological features, morphological structure, and metabolic processes in biological materials. When optically absorbent objects (absorbent materials) inside the tissues are bombarded with a brief (nanosecond) pulse laser, the PA effect occurs. The target absorbs the pulse energy with the help it heat, resulting in a temporary transient temperature increase accompanied by a local sound pressure rise due to thermoelastic contraction [1].

The image of photoacoustic is a new hybrid imaging technology that uses both ultrasonic and optical contrast. Optical imaging has been shown to discover and describe a variety of vascular abnormalities in the breast because of its capacity to discriminate hypoxic blood pools. PAI may potentially add significantly to dynamic or static difference investigations, seeking for vascular abnormalities and breast cancer screening, in identifying several vascular irregularities now found by magnetic resonance, with gadolinium-based contrast compound injections and high expense and difficulty. Numerous reports have described the application of PAI to breast cancer detection. The quantity of ionic water in the breast tissues was responsive towards this microwave-induced thermo-acoustic photography. Furthermore, the company achieves amazingly comprehensive breast angiogram on one individual employing PAVI at a relatively high rate of 5 MHz and strong focal gain of tiny ultrasound (US) components on a rotating disk. For 3-D screening mammography, researchers developed the Twente method, which uses a planar 2-D array with 590 components read out by a single processor stream [5].

Ultrasound sensors outside of the tissues identify changes in pressure traveling as ultrasound waves, which are referred to as original data (Figure 1). These statistics collect details about the absorbers' intrinsic acoustical and visual capabilities, as well as noisy data resulting from electromagnetic disruptions. The collected data is then analyzed (known as signal processing) in order to extract the necessary PA signals from the chaotic ambient and use it to rebuild a PA visual. The internal structures and accompanying function of the tissues targeted area are depicted in these photos. For PA scanning, many picture reconstruction techniques have been explored, each of which could be understood as an acoustic inversion source issue. The acoustic parameters of the object of interest are assumed to be homogeneous in traditional PA picture imaging techniques [6].

Nevertheless, in actuality, the cellular substrate is the heterogeneity, with sound speed and density dispersion that differs regionally. This causes acoustic distortion (i.e., amplitude reduction, signal widening, and mode transformation), which ultimately enhances low-frequency vibrations and impacts narrow wavelength, which correlates to nanostructure and sharp corners. As a result, image resolution, which is one of PAI's key contributions, is sacrificed. Furthermore, considerable distortions and artefacts are introduced due to varying acoustic dispersion. Although advances in PA iterative reconstruction techniques that can adjust for changes in acoustical qualities have been made, additional picture augmentation in terms of postprocessing is still required [7].

Many illness detection techniques use deep learning, which is enhancing machine academic performances in the sector. A feedforward neural net called a multilayer perceptron (MLP) is a recent innovation for use in deep learning to recognize and analyze various malignancies. DL has been utilized as stacked denoising autoencoders (SDAE) to convert high-dimensional information speckle noise to low-dimensional information for the classification of breast, according to a previous work. In another study, the job of gene connection prediction in a supervised scenario was completed using a fresh strategy called convolutional neural network for co-expression (CNNC), which was suggested and applied [8]. The extraordinarily huge scale of diseased data, which could be in the gigapixels, presents a barrier while using deep convolutional neural networks (DCNNs). Research suggested using tiny bits of the high accessibility for a CNN in breast cancer separation to solve this problem. To train the CNN, the initial whole slide image (WSI) was split into multiple chunks, with the ultimate decision taken by aggregating the findings for every region. To aggregate the patch-wise outcomes, other decision procedures were applied; nevertheless, they all showed similar results, and none of them outperformed the separate results. The researcher increased the performance of patch-based CNNs by combining the patch-wise results with a support vector machine (SVM) [9].

Since their adaptability, intelligent optimization techniques have been widely employed in many study domains. They are generated by mimicking or disclosing some natural events. Because of its accessibility and versatility, the PSO (particle swarm optimization) method has indeed been successfully utilized for classification tasks. Particle swarm, on the other hand, is simply included in the local optimum. Furthermore, the ABC (artificial bee colony) algorithm has strong international resolution and a wide range of applications. ABC, on the other hand, fails miserably at exploiting. In tackling complicated problems, using a single optimization method has the drawbacks of low precision and poor generalization ability. PSO and ABC are integrated into this study to further investigate the use of intelligent optimization in bioinformatics, which means the ability of exploiting and investigation are merged for binary data [10]. Various scholars have recently applied deep learning algorithms with/without domain adaptation for object detection, microcalcification, and bulk recognition. To avoid this need for massive data in training, ensemble learning uses information from those other areas in the shape of pretrained model extraction of features levels. In this version, the system utilizes data to fine-tune its training parameters or the region of interest's uttermost classification layer. For assessment detection, researchers used a context-sensitive deep convolutional neural network. For mass categorization, researchers used intensity information and deep features generated from a deep convolution neural network (CNN) [11].

## 2. Related Works

Prostate cancer is among the most frequent cancers in men, and it is the third highest cause of cancer mortality in the world. Already extensively explored diffusion-weighted magnetic resonance imaging (DWI) was an incorporated aspect of computer-aided detection (CAD) methods for reliable prostate cancer detection. To achieve the great results from deep convolutional neural networks (CNNs) in machine learning computer vision applications classification and extraction, various CNN structures have been progressively being evaluated in the clinical imaging scientific community as convincing results for developing more precise cancer detection CAD tools. DWI is an MRI series that assesses tissue's responsiveness to Brownian motion and has already been identified as a viable imaging tool for PCa identification. The DWI imaging is often produced using various *b* values, resulting in varying signal intensity that indicates the quantity of liquid diffusion in the tissues and could be utilized to calculate ADC and calculate high *b*-value imaging. Researchers devised and deployed an automatic CNN-based process for detecting clinically relevant prostate cancer (PCa) for every individual and every axial DWI imaging throughout this study. The fundamental problem of this study is that like CAD publications, the material is fundamentally skewed; individuals that have an indicator of prostate cancer have been sent to an MRI. As a result, the information does not accurately represent the population. Furthermore, the information labels were dependent on biopsy regions that are established by physicians. In other words, depending on radiological data, slices without a biopsy were considered to be negative. The positive segments, on the other hand, are predicated on pathology (biopsy) findings [12].

The extensive study into healthcare clinical systems is providing abundant opportunities for computational systems to develop the most cutting-edge advancements. Such advancements were contributing to more accurate healthcare technology systems that include computerized detection of health-related issues. One of the most essential health studies was conducted in order to forecast cancer, which could take several kinds as well as damage various sections of the organism. Pancreatic cancer is among the most common cancers that are projected to be incurable. These could not be addressed well once diagnosed and, throughout most situations, are determined to be unpredictable because it is located in the abdomen underneath the stomach. As a result, advances in clinical knowledge are leading to the development of automation processes that could detect the detection and screening and provide appropriate diagnosis and treatment if they are detected. Deep learning is one such topic that has expanded its study into diagnostic imaging, automating the procedure of detecting a patient's condition while combined with a collection of equipment such as CT/PET scan devices. The convolutional neural network (CNN) framework has been used in the study to predict cancer images of the pancreatic that is integrated with the Gaussian distribution with EM method to identify the main characteristics out from computed tomography as well as assumes the proportion of cancer spread in the pancreatic using the threshold parameters as indicators. However, the collection is restricted in this study because fitting a Gaussian model involves a huge number of factors, as well as a huge amount of data and many repetitions [13].

The irregular and fast development of breast cells causes breast cancer. Early detection could lead to more straightforward and efficient therapy. Although surgeons have a tough time distinguishing diseased cells from healthy tissues for identification, a lump in the breast seems to be a key accurate marker of breast cancer. In the latest days, the advancement of computer-aided identification processes results in nondestructive as well as effective cancer diagnostic approaches. Throughout this study, a complete technique for locating the malignant zone in a mammography image is proposed. Image distortion removal, optimized image segmentation using a convolutional neural network, a grasshopper optimization algorithm, as well as optimized feature retrieval and feature selection using the grasshopper optimization algorithm are all used in this technique, which improves accuracy while lowering computational costs. The simulated outcomes are then compared using 10 various state-of-the-art techniques to inspect the suggested process performance, as well as the findings, which have been implemented in the Mammographic Image Analysis Society Digital Mammogram Database and the Digital Databases for Screening Mammography breast cancer data sets. The GOA, on the other hand, has several disadvantages, including a slow convergence speed and a proclivity for dropping into locally optimal solutions. In addition, the fundamental linear convergence factor enables the exploratory and exploitative operations to be imbalanced [14].

Prostate cancer could range in severity from low-risk ones that could be managed with close monitoring to high-risk stages that could be fatal if left untreated. The development of noninvasive as well as medically significant technologies for screenings, detecting, prognostic, and disease surveillance, including therapy effectiveness predictions is crucial. Researchers concentrate on significant breakthroughs as well as prospective activities required to propel therapeutic innovations throughout this field of urinary biomarkers and therapeutic for detection of cancer as well as prognostication in this analysis. An overview of the published studies on urine biomarkers indicating prostate cancer is presented. Researchers assess the benefits and drawbacks of a range of methods that differ in survey methods as well as benchmarks evaluated; researchers discuss noted urine samples for prostate cancer throughout the terms technically, methodically, and with clinical parameters; and researchers offer their thoughts on important aspects in establishing an experiment-based urine for prostate cancer. There is a long history of research on urination as a collection of biomarkers for prostate cancer, which has produced a number of urine samples in medical usage today. Theoretical and methodological advancements in the field would aid in the development of new urine samples, which could cause significant changes in the therapeutic paradigms for prostate cancer diagnosis and treatment. Certain times utilizing biomarkers will not help; since leading an experiment to differentiate biomarkers, it is dynamic to appropriately plan the investigation. About 80–90% of all biomarker populace throughout the previous 20 years has not and cannot be repeated, and the fundamental explanation that biomarkers vanish is that these examinations are not planned as expected [15].

Accurate diagnosis of thyroid nodules could reliably identify cancer incidence and guide tailored care. Researchers present a new multimodal MRI-based computer-aided diagnosis (CAD) approach for determining whether thyroid nodules are cancerous or normal. The suggested CAD is built on a revolutionary textural modeling structure depending on convolutional neural networks (CNNs). This technology allows a threefold advantage. To begin, the method is revolutionary at the time to use a CNN to simulate thyroid cancer using apparent diffusion coefficient (ADC) maps with T2-weighted MRI. Secondly, it acquires distinct textural properties for every source, allowing it to retrieve complicated texture patterns from both modalities at the same time. Furthermore, the suggested system combines several scanning gathered into the deep learning procedure utilizing high variability of the customizable diffusing gradients parameter utilizing various systems for every input. As a result, the suggested system would allow for the acquisition of more complicated radionics, as well as the visualization of complex surfaces following the acquisition. The suggested approach was tested utilizing information from 49 patients who had pathologically verified thyroid nodules. The suggested system's efficiency has also been evaluated to modern CNN models and also a variety of machine learning (ML) systems, which include handcrafted characteristics. However, there seem to be significant constraints that must be resolved before too many medical studies may be conducted. Because the number of samples in the analysis is minimal, the findings also imply the pattern, which is presented in this group. In order to examine the consistency of texturing between groups, it needs to apply the algorithm to some other cohort with a larger number of patients. To adequately capture the complete range of thyroid cancer, additional samples were gathered [16].

Thyroid nodules are malignant or benign tumors of liquid-filled or hard tumors that grow within the thyroid gland. The goal would be to see if incorporating the mentioned aspects of the thyroid imaging reporting as well as data system (TI-RADS) into a software system might help radiologists make better decisions. Researchers created a computer-aided disease diagnosis that has been connected to multiple-instance learning (MIL) and focused on benign-malignant classifications throughout this work. The Universidad Nacional de Colombia provided the data. There must have been 99 cases in total (33 benign and 66 malignant). For picture preprocessing including segmentation, the median filter with image pattern classification has been used in the work. Seven ultrasonography picture features have been extracted using the grey-level co-occurrence matrix (GLCM). The information was split into two sets: 87% training and 13% verification. On the basis of accuracy, sensitivity, and specificity, researchers evaluated the artificial neural network (ANN) as well as support vector machine (SVM) classification techniques. The thyroid nodule's benign or malignant status has been the assessment instrument. Researchers also created a graphical user interface (GUI) to present image attributes that might assist physicians in making decisions. The reliability of ANN and SVM was 75% and 96%, respectively. Overall success factors showed that SVM outperformed most other algorithms, with increased precision, sensitivities, and precision. MIL appears to have promising outcomes in the identification of thyroid cancer, according to the findings. Once the classification algorithm could be used in practice, more validation with additional information is necessary [17].

Modern prostate-specific antigen (PSA) depending on screened has a large rate of false negatives and positives, many of that have unfavorable effects. The National Cancer Institute's Prostate, Lung, Colorectal, and Ovarian Cancer Screening Trial delivered us with a database of 36,952 individuals. Researchers distributed the process into various sets: those that had high-risk prostate cancer, those who had low-risk prostate cancer, and those who did not have prostate cancer. Researchers developed a pipeline to manage unstable data as well as presented preparation strategies for these data sets. Researchers looked at how well different machine learning techniques predicted high-risk prostate cancer. The proposed pipeline, which uses traditional scalability, the SVMSMOTE sampling approach, with AdaBoost for computer vision, could attain 91.5% accuracy. The reliability of such an approach was then assessed using the speed of adjustment of PSA, age, BMI, and filtering by race. Researchers discovered that integrating the speed of adjustment of PSA with age in the analysis raised the model's area under the curve (AUC) by 6.8% although BMI, as well as race, seemed to have no impact. Researchers developed a machine learning algorithm for the prostate screenings component of the National Cancer Institute's (NCI's) Prostate, Lung, Colorectal, and Ovarian Cancer Screening Trial (PLCO) in this study. Although specific types of estrogens were distinguished, the picture became more complex and difficult, because the recognition of classical estradiol receptors ( and ) has a different effect on the development of prostate cancer and the current paucity of models of prostate cancer and its covariates due to the conflicting nature of the results makes the involvement of estrogens (i.e., regardless of whether participants increase or decrease the prevalence of prostate cancer) a difficult question to answer [18].

Thyroid cancer is among the most frequent cancers, including both men and women experiencing a rise in the estimated incidence. The existing gold standard for diagnosing thyroid malignancies is ultrasound-guided fine-needle extraction; however, the findings are erroneous, resulting in unneeded biopsies and procedures. Researchers investigated the use of multiparametric photoacoustic (PA) testing in conjunction with the American Thyroid Association (ATA) guidelines to decrease the number of unnecessary biopsies (ATAP). Researchers used in vivo multispectral PA imaging on thyroid nodules among 52 individuals, 23 of whom had papillary thyroid cancer (PTC) and 29 of whom had benign thyroid nodules. Researchers computed haemoglobin oxygen intake in the nodule region using multispectral PA data and then identified the PTC with benign nodules using a multiparametric approach. The multiparametric assessment of multispectral PA signals was able to categorize PTC tumors, according to statistical studies. Integrating PTC's photoacoustically suggested likelihood with the ATAP resulted in a novel scoring technique with 83% sensitivities and 93% accuracy. This is the first statistically significant multiparametric assessment of multispectral PA data of thyroid nodules. The findings indicate that perhaps the suggested improved ATAP grading could help clinicians analyze thyroid cancer for fine-needle extraction biopsies, minimizing needless biopsies as a conceptual design. However, every photodetector in multispectral screening targets a wide area, and any light outside the associated wavelength zone is ignored. It has a negative impact on sensitivity, especially as the amount of frequency channels increases [19].

## 3. Methodology

A unique PS-ACO-RNN approach to recognizing and classifying cancer using multispectral photoacoustic imaging was developed in this work. The developed PS-ACO-RNN approach involves several steps, including bilateral filtration based on processing, segmentation based on LEDNet, feature extraction based on PS-ACO, and classification based on RNN. The following sections explain how each module of the PSO-ACO-RNN approach works in detail.  Figure 2 depicts the basic flow diagram for the recommended approach.

### 3.1. Data Collection

The multispectral photoacoustic test image is collected from the online database of academic torrents cancer data sets (https://academictorrents.com/browse.php?search=cancer&c6=1). The data sets are validated to 70:30 ratios for training and testing of the specimens. Due to the inconsistency in the data collection, most of the data are not uniform, and it changed from 20 × 64 × 200 pixels to 64 × 64 × 200 pixels. The *X*- and *Y*-directional equalization was achieved by enlarging the size to 64 × 64 pixels and using linear interpolation.

### 3.2. Data Preprocessing

The bilateral filtration approach is used as an image processing technique in this research. It gives smoothness to the images without affecting their edges using nonlinear amalgamation of the closed values of the image. The given strategy is simplest, localized, and unknown. Depending on the geometric proximity and photometric similarities, it integrates the grey levels. It selects the domains closest to the value range and distance values. CIE-Lab uses two-page filtration for basic perceptual parameters in the space color, retaining the edges and smoothing the color to suit the human viewing, unlike filtering in three independent color bars [20].

### 3.3. Image Segmentation

LEDNet uses an encryption-decryption mechanism that uses an asymmetric hierarchical structure in which encryption results in a reduced feature map which is modified by the APN, which optimizes the feature map to suit the input resolution. In addition to the SS-nbt unit, downsampling is done with two parallel results stacked on a solitary 3 × 3 convolution with max pooling and straight 2. The downsampling provides much in-depth networking to capture the contexts while minimising computing time. Furthermore, the extended convolutional process allows the infrastructure to capture a larger acceptance domain, leading to increased accuracy. This method was developed to improve performance in terms of processing costs and variables using a larger kernel size.

The decoded design APN for spatial assessment executes uses spatial-wise focuses designed by the attention process. The APN accepts a pyramid focus component, which expands the responsive domain by combining elements from three distinct pyramid sizes. It first uses the 3 × 3, 5 × 5, and 7 × 7 convolution with straight 2. Then, pyramid architecture combines information from multiple dimensions one after the other, perfectly integrating the neighboring dimensions of the context. Using a larger kernel size does not add system load, as the upper-level feature map has a lower resolution. Following that, a 1 × 1 convolution was applied to the coded effect, and there was a pixel-wise multiplication feature map by the pyramid focus component. Design a global average pooling branch to integrate the previous core of the overall environment to increase performance An upsampling device was eventually used to match the resolution of the input images [21].

### 3.4. Extracting Features

During the process of extracting features to detect lesion sites in multispectral photoacoustic imaging, the segment image is sent to the PS-ACO approach.

### 3.5. Particle Swarm Optimization

It is a biologically induced mechanism that seeks the optimal method in a straightforward way at the solution location. The selection of random images, *N*, is used to start the process. Positioning the *n*^th^ image as a point in the *V*-dimensional space indicates the number of “*V*” variables used to identify it. Each image tracks three data during the “*n*” process: its current location (Cn), the optimum level reached in previous cycles (On), and its flying speed (Fn). The codes for these three levels are as follows:

  Current location Cn = (*C*_*n*1_, *C*_*n*2_, *c*_*n*3_,…, *C*_*nv*_)
  Optimum level reached in previous cycles *O*_*p*_ = (*O*_*n*1_, *O*_*n*2_, *O*_*n*3_,…, *O*_*nv*_)
  Flying velocity *F*_*n*_ = (*F*_*n*1_, *F*_*n*2_, *F*_*n*3_,…, *F*_*nv*_)

The best image (gbest) positioning (Pgbest) is rated the best fit for all images in each period (cycle). As a result, each image adjusts its speed to get very close to the best image gbest, and new velocity is given below.

(1) $$\begin{array}{c} \text{New}F_{n}=\delta \times \text{current}F_{n}+l_{1}\times \text{rand}\left(0,1\right)\times \left(O_{p}-C_{n}\right)+l_{2}\times \text{rand}\left(0,1\right)\times \left(O_{p}-C_{n}\right), \end{array}$$

where *l*_1_ and *l*_2_ represent two significant constants called learning variables; rand (0, 1) refers to two random features in the range [0, 1], the potential for greater change in particle velocity over *V*_max_; and *δ* is the inertia weight used as an improvement to handle the influence of the previous history of velocities at current speeds.

### 3.6. Ant Colony Optimization (ACO)

The second technique for short-scale development uses an optimization function to test one dimensionality, reliability based on saturated components, potential discrimination across capacity distribution, and changes in relationships for covariates. Ant colony optimization generates a large number of ant colonies looking for the optimal characteristics parallel to a particular discriminant problem in the high-dimensional spectrum variable space.

The ACO algorithm performs a series of cycles consisting of the following three essential concepts: the universal pheromone is used to create images that are assigned to trace spectral elements with probability; the efficiency of each image is measured; and the trace evolution constants of global pheromones and the classification of images are updated using performance. All three procedures are repeated to obtain global optimal forecast performance. A change probability model is used to give spectral parameters for image clusters.

(2) $$\begin{array}{c} Pn\left(t\right)=\frac{{\left(\mu n\left(t\right)\right)}^{\alpha \;}\varphi n^{\beta }}{\sum_{n}{\left(\mu n\left(t\right)\right)}^{\alpha }\varphi n^{\beta }}, \end{array}$$

where *µn* (*t*) is the quantity of pheromone for the *n*^th^ spectral parameter at period *t*, ф*n* is local data, and *α* and *β* are the weighting specifications for the pheromone and local information, respectively.

### 3.7. Hybrid Approach (PS-ACO)

In the case of global optimization techniques, the hybrid universal optimization system based on recombination is the most widespread. The simulated ant colony method and particle swarm optimization are two of these methods. Although ACO has a strong ability to detect global optimization, the global best solution is not used immediately because it is stored in every iteration; unlike particle swarm optimization (PSO), the global best solution can be used in every iteration. The entire process of the hybrid approach is represented in Figure 3.

This compound was used in the study to create a new solution called “FinalBest.” For PSO, FinalBest is the gbest, while for ACO, it is the neighbor of spectator ants. To create FinalBest, the optimal values for PSO's gbest and ACO's best solution are calculated, and the probability selection for both results is calculated using these fitness values.

The probability of the best solution for ant colony optimization is represented below:

(3) $$\begin{array}{c} P_{\text{best}}=\frac{{\text{fitness}}_{\text{best}}}{{\text{fitness}}_{\text{gbest}}+{\text{fitness}}_{\text{best}}}. \end{array}$$

The probability of the best solution of the particle swarm optimization is represented below:

(4) $$\begin{array}{c} P_{\text{gbest}}=\frac{{\text{fitness}}_{\text{gbest}}}{{\text{fitness}}_{\text{gbest}}{+\text{fitness}}_{\text{best}}}. \end{array}$$

The probability of best solution of hybrid optimized final outcome is represented below:

(5) $$\begin{array}{c} {\text{Final}}_{\text{best}}=\left\{\begin{array}{c} {\text{best}}_{n},\text{if }\left(r<P_{\text{best}},\right.\\ {\text{gbest}}_{n}\text{, otherwise.} \end{array}\right. \end{array}$$

This study describes the relationship between particle mass optimization in the hybridization of ACO and PSO and artificial ant colony. The construction of a new variable named “FinalBest” is the result of the interaction between these two methods. As mentioned earlier, this parameter helps increase the exploitation capacity of the ACO by directly utilizing the best data in the world, as well as the ability of the PSO to remove the local minima.

### 3.8. Image Classification

The PS-ACO-RNN model can be utilized to diagnose and classify cancer using ultrasound images at the end of the procedure. In the traditional NN, all input and outputs are considered to be autonomous of each other. However, this assumption is incorrect in many applications, especially in applications that use serial data such as speech recognition functions. RNN, unlike a traditional NN, delivers output based on the previous state and performs a similar function from time to time to subsequent components. In other words, a memory holds previously calculated data with the help of RNN. RNN is a kind of neural network that is often used for language modeling and has been shown to be very effective in cancer classification tasks. Data travels only one way from the layer of input to the output, passed by the hidden layer. The information has been transferred in a straight line via the network, not passed by the similar node twice.  Figure 4 depicts the RNN classification and its outcomes PS-ACO-RNN cancer detection mechanism procedure mentioned below in Algorithm 1..

## 4. Result and Discussion

The validating performance of the PS-ACO-RNN approach is carried out by using the multispectral photoacoustic image. In this, 70% of data are used for training, and the remaining 30% of data are used in the testing process.

The recurrent neural network parameters are updated using gradient descent in the learning process. The learning rate is initialized at the rate of 0.01 when the network is trained and the exponential of decay is about 0.1 for each epoch, which is given in Figure 5. The set of hyperparameters such as number of layers, size of the bilateral filter, fully connected layer, learning rate, and activation function are used in this system for selecting the random start of the proposed system.

In the proposed technique, out of three prostate, it can be able to detect three cancers, and out of two thyroid cancer, one cancer can be detected. The capability of detecting the cancer in the MPA data set is given in Table 1.

The ROC analysis of PS-ACO-RNN is demonstrated in Figure 6, using the training and testing data set of MPA. It exposed that the proposed system provided enhance region of the curve by about 98.4% on the training and testing data set.

The accuracy of training and testing a data set using the PS-ACO-RNN technique and its outcome is illustrated in Figure 7. The accuracy of testing is enhanced compared to the accuracy of training a data set using the proposed technique. The accuracy of the concentrated value is based on the number of epochs.

The loss of training and testing a data set using the PS-ACO-RNN technique using the MPA data set is illustrated in Figure 8. It is analyzed that the validation loss of the training is reduced using this approach, and based on the number of epochs, the loss value is saturated.

The effectiveness metrics of the proposed method is compared with the existing technique such as recurrent neural network, convolution neural network, support vector mechanism, and *k*-nearest neighbor technique illustrated in Table 2, and the graphical representation is shown in Figure 9. It is analyzed that the performance of the proposed PS-ACO-RNN technique is better compared to other techniques.

## 5. Discussion

The modality of the medical image is analyzed using photoacoustic imaging. The single tissue information such as thyroid and prostate of the clinical data set is sufficient because the deep learning technique requires a greater number of samples for more efficient recognition. In this work, multispectral photoacoustic imaging with mixed prostate and thyroid is used to train the proposed network. The photoacoustic image is used for extracting the features of cancer from different tissues.

The recurrent neural network is proposed, which is more robust and provides a more accurate classification for detecting cancer. The RNN can easily extract the feature for decreasing the problem of detecting cancer tissues. The particle swarm and ant colony optimization is used with the RNN network to enhance the performance in detecting the cancer tissue in MPA imaging.

## 6. Conclusion

This work incorporates a unique PS-ACO-RNN technique for diagnosing and classifying cancer using ultrasound images. Based on bilateral filtration processing, LEDNet for separation, PS-ACO for feature extraction, and RNN-based classification are all part of the proposed PS-ACO-RNN approach. Continuous simulations using the benchmarking database can be used to show the best results of the PS-ACO-RNN model. Extensive comparative findings proved that the PS-ACO-RNN strategy outperformed all other approaches. Consequently, the PS-ACO-RNN model can be used to classify cancer using ultrasound images as a useful tool. Advanced DL techniques may be used in the future to improve cancer classification accuracy.

## Figures and Tables

**Figure 1:** Basic flow on photoacoustic imaging.

**Figure 2:** Basic diagram for the recommended approach.

**Figure 3:** Entire processing of PS-ACO-RNN algorithm.

**Figure 4:** RNN-based cancer classification.

**Figure 5:** Epoch with learning rate decay.

**Figure 6:** Generated ROC curve.

**Figure 7:** Training and testing accuracy using PS-ACO-RNN technique.

**Figure 8:** Training and testing loss using PS-ACO-RNN technique.

**Figure 9:** Performance metric of proposed PS-ACO-RNN technique with other current approaches.

**Algorithm 1:** PS-ACO-RNN cancer detection mechanism.

**Table 1:** Performance metrics of the proposed system using MAP data set.

	Precision (%)	Recall (%)	*F*-measure (%)	Support
Cancer	100	80	89	11
Normal	92	100	96	5
Average	94	94	94	16

**Table 2:** Performance comparison of the proposed technique with the existing technique.

Method	Accuracy	Precision	Recall	*F*-measure	AUC
Proposed PS-ACO-RNN	98.6	98	94	98	
RNN [22]	97.3	98	97	98	95
CNN [23]	95	80	77	78	87
SVM [24]	88	78	85	76	92
KNN [25]	89	84	76	90	98

## Data Availability

The data used to support the findings of this study are included within the article.
